This article has been retracted.

# Clinical Effect of Hufu Copper Scraping on Shoulder-Hand Syndrome after Stroke

**DOI:** 10.1155/2022/9165141

**Published:** 2022-08-25

**Authors:** Lianyi He, Xinyu Chen, Yuejuan Zhang

**Affiliations:** ^1^Department of Cadre Health Care, The First Hospital of Hunan University of Chinese Medicine, Changsha, Hunan 410007, China; ^2^Department of Cardiovascular Medicine, The First Hospital of Hunan University of Chinese Medicine, Changsha, Hunan 410007, China; ^3^Hospital of Hunan University of Chinese Medicine, Changsha, Hunan 410007, China

## Abstract

**Objective:**

To explore the clinical effect of Hufu copper scraping on shoulder-hand syndrome after stroke.

**Methods:**

A total of 60 patients with shoulder-hand syndrome after stroke admitted to the First Affiliated Hospital of Hunan University of Traditional Chinese Medicine were enrolled between January 2020 and June 2021. According to the random number table method, they were divided into the control group (*n* = 30) and the intervention group (*n* = 30). The control group was given routine rehabilitation intervention, while the intervention group was additionally given Hufu copper scraping. The intervention effect, occurrence of adverse reactions during the intervention, pain, swelling degree of affected hands, serum calcitonin gene-related peptide (CGRP), substance P (SP), and Barthel index before and after 2 months of intervention were compared between the two groups.

**Results:**

After intervention, the total response rate of the intervention group was significantly higher than that of the control group (96.67% *vs* 80.00%) (*P* < 0.05). After intervention, the score of the visual analogue scale (VAS) and water displacement in the intervention group were lower than those in the control group (*P* < 0.05). After intervention, levels of CGRP and SP in the intervention group were lower than those in the control group, while the Barthel index was higher compared to the control group (*P* < 0.05).

**Conclusion:**

The intervention effect of Hufu copper scraping is good, which can promote the recovery of related symptoms, relieve pain and swelling of affected hands, downregulate levels of disease-promoting markers, and accelerate recovery of related function in patients with shoulder-hand syndrome after stroke.

## 1. Introduction

Shoulder-hand syndrome, also known as reflex sympathetic dystrophy, complex regional pain syndrome type I, is a common complication of stroke patients, and mostly occurs 2 weeks–3 months after cerebral infarction or cerebral hemorrhage. It is manifested as pain in the shoulder, hand, wrist, other parts of the upper limb on the affected side, limited joint activities, obvious atrophy of skin and muscles in the late stage, and in severe cases, it can lead to complete loss of hand function [1]. The most effective means of shoulder-hand syndrome is early prevention so that the affected limb can maintain its functional position, strengthen the passive and active activities of the affected limb, especially the shoulder and hand, and relieve the pain of the patient. Through proper physical therapy and early rehabilitation training, the disease progression of shoulder-hand syndrome can be controlled and the functional rehabilitation of affected limbs can be promoted [2]. At present, the clinical treatment methods for shoulder-hand syndrome mainly include drug therapy, rehabilitation therapy, and surgical therapy, among which the internal and external treatment schemes of traditional Chinese medicine have good therapeutic effects on the disease (TCM) [3]. Gua sha (scraping) is a nondrug characteristic therapy of TCM. By using special scraping tools such as friction, scraping, and other techniques to produce benign stimulation to meridians and acupoints, it achieves the effects of relaxing tendons and promoting blood circulation, removing blood stasis, expelling pathogens, and curing diseases [4]. Some studies have confirmed that scraping has important application value in promoting the functional recovery of patients with poststroke shoulder-hand syndrome [5, 6]. Hufu copper scraping therapy is a branch of traditional scraping therapy, which uses special instruments and has a stronger effect. In this study, the Hufu copper Bianstone made of brass will be used for scraping therapy for stroke patients with shoulder-hand syndrome to explore its clinical effect and to provide a certain basis for clinical-related research. The report is as follows.

## 2. Research Objects and Methods

### 2.1. Research Objects

A total of 60 inpatients with shoulder-hand syndrome after stroke in the First Affiliated Hospital of Hunan University of Traditional Chinese Medicine from January 2020 to June 2021 were selected. The numbered patients were divided into the control group (*n* = 30) and the intervention group (*n* = 30) by random number table method. Among them, there were 21 males and 9 females in the control group, aged 18–65 years, mean (45.43 ± 8.57) years old, disease duration from 2 weeks to 6 months, mean (3.48 ± 1.17) months, etiology; there were 12 cases of arteriosclerosis type, 6 cases of cardiogenic type, 6 cases of arteriole occlusion type, and 6 cases of other reasons, the affected side; 16 cases in the left hemisphere and 14 cases in the right hemisphere; there were 18 males and 12 females in the intervention group, aged 18–65 years, mean (46.29 ± 8.73) years old, disease duration from 2 weeks to 6 months, mean (3.73 ± 1.05) months, etiology; there were 14 cases of arteriosclerosis type, 5 cases of cardiogenic type, 6 cases of arteriole occlusion type, and 5 cases of other reasons, the affected side; 17 cases in the left hemisphere and 13 cases in the right hemisphere. There was no significant difference in baseline data between the two groups (*P* < 0.05), which was comparable. This study was approved by the hospital ethics committee.

### 2.2. Diagnostic Criteria

The diagnostic criteria of ischemic stroke include [7] acute onset, focal neurological deficits (one side of the face or limbs weakness or numbness, language disorders), a few facial nerve functional deficits; the responsible lesions or symptoms and signs appear on imaging for more than 24 hours; exclude nonvascular diseases; brain CT excluded cerebral hemorrhage.

TCM diagnostic criteria for ischemic stroke include clinical manifestations: fainting of consciousness, hemiplegia, strong tongue, or even no language, limbs withered and useless; headache, dizziness, changes in pupils and spirits, not blinking eyes, choking when drinking water, and unsteady walking; onset mode: acute onset, most onset is in a quiet state, progressive aggravation, or a history of repeated similar symptoms. A small number of patients may have a sudden onset, rapid disease progression, and dizziness; incentives before the onset: every time, it is induced by emotional injury, improper diet, and impermanence of daily life. There are often aura symptoms, such as dizziness, headache, tinnitus, sudden transient difficulty in speech or numbness of limbs, and blurred vision; age of onset: takes place in people who are more than 40 years old. With the above clinical manifestations, combined with the form of onset, incentives, aura symptoms, and age, the diagnosis can be made. Combined with imaging studies (head CT/MRI), the diagnosis can be confirmed. Let us look into the diagnostic criteria of shoulder-hand syndrome [8]. In accordance with the symptoms, it is divided into three stages, the first stage is swelling of the hands, color changes, and painful movement disorders in the shoulders and hands; stage II: painful movement disorders of the shoulders and hands are relieved, swelling and color changes are partially relieved or completely disappeared, and muscle atrophy begins; stage III is dystrophic changes in the hands and shoulders, with obvious muscle atrophy, limited joint movement, and contractures.

### 2.3. Inclusion Criteria

The inclusion criteria were as follows: selected patients also meet the diagnostic criteria of Chinese and Western medicine for ischemic stroke patients with stage I shoulder-hand syndrome; the first onset was confirmed by head CT or MRI, and the course of the disease was in the recovery period of 2 weeks to 6 months; age 18–65 years old; vital signs are stable and can cooperate with examination and treatment; patients or their family members gave and signed the informed consent form.

### 2.4. Exclusion Criteria

The exclusion criteria were as follows: those who are combined with the liver and kidney failure, respiratory failure, heart failure, blood system, and other diseases; those who are unable to cooperate due to aphasia or severe cognitive dysfunction; those who have a history of mental illness or dementia; those who are allergic to the oil scraping or have a history of severe allergy; and patients with poor compliance and readmission.

### 2.5. Suspension and Rejection Criteria

① Those who have other serious diseases during the intervention process; ② intolerance or treatment site infection and other adverse reactions occurred during the intervention; ③ patients with recurrence or serious complications during the intervention; ④ those who could not complete the intervention due to insufficient treatment course withdrawal or death.

### 2.6. Methods

Both groups of patients were given secondary vascular preventive treatment according to the “Guidelines for the Prevention and Treatment of Cerebrovascular Diseases in China” [9], and symptomatic treatment was given according to the patients' underlying diseases, including antiplatelet aggregation drugs, plaque stabilization, antihypertensive drugs, and blood sugar control. For treatment, avoid the use of nonsteroidal anti-inflammatory analgesics. When the patient is sitting or standing, we use the shoulder strap to support the patient's upper limb on the affected side, and place the affected limb in a good position when lying down. Both groups of patients were given routine rehabilitation therapy, good limb placement, exercise therapy, occupational therapy, physical factor therapy, and so on.

The control group received routine rehabilitation treatment. Each rehabilitation treatment time was 40 minutes, 2 times a day, 5 days per week, and the intervention period was 2 months. The specific method was given according to the patient's condition. For example, properly train the patient to rotate the affected shoulder and bend the elbow joint, taking the patient's conscious feeling as the degree; Medical staff help to move the affected limb, conform to the movements of the joints of the shoulder, elbow and wrist, so as not to cause pain.

On the basis of the control group, the patients in the intervention group were given Hufu Copper Bianstone scraping, 1 time a week, 1-2 hours each time; 4 weeks as a course of treatment, a total of 2 courses of treatment. The patient is placed in a supine position, the upper limbs are exposed, kept warm, and applied an appropriate amount of scraping oil on the skin surface. The details are as follows: (1) Scraping device and medium: the scraping device used is the Hufu Copper Bianstone made by Wenshatang, and the oil scraping is the special scraping oil made by Wenshatang. After scraping, clean the scraping board with hand sanitizer, then rinse with clean water, dry with a soft cloth, and send it to the supply room for autoclaving and disinfection. If the scraping device is contaminated with blood or body fluids, the contaminants should be removed in time, and then soaked in a disinfectant containing 2000 mg/L–5000 mg/L of effective chlorine for more than 30 minutes, rinsed with clean water, and sent to the supply room for autoclaving and disinfection after drying. (2) Meridian and acupoint selection; ① Meridians: mainly Yangming meridian, Du meridian, and bladder meridian of Foot Taiyang, plus the three Yang and three Yin meridians on the inside and outside of the hands and feet, and combined with some parts of the patient's symptoms; ② Acupuncture points on the back: Dazhui (DU14), Dazhu(BL11), Gaohuang(BL43), and Shentang(BL44); ③ Acupuncture points for the head and face: Baihui (DU20), Yintang(DU29), Jiache(ST6), and Dicang(ST4); ④ Acupuncture points for upper limbs: Jianyu(LI15), Quchi(LI11), Shousanli(LI10), Waiguan(SJ5), Lieque(LU7), and Hegu(LI14) on the Yang side, Jiquan(HT1), Chize(LU5), Quze(PC3), Daling(PC7), and Neiguan(PC6) on the yin side. (3) Gua sha method, first open the four acupuncture points, namely Dazhui, Dazhu, Gaohuang, and Shentang to stabilize the lower Jiao, then scrape the Du meridian on the back and the bladder meridian of Foot Taiyang, and then scrape the third hand on the outer side of the upper limb on the healthy side in turn. The Yang meridian runs through the part of the hand, the Sanyin meridian on the inner side of the upper limb runs through the part of the limb until the end of the limb, the affected side is first acupunctured on points with fingers, and then scraping is carried out. Scraping strength depends on the patient's tolerance, rather than forcing scraping on the spot. (4) Notes: ① the treatment time for the first-time scraping patients should not be too long, and the patients should be frequently asked about their feelings, and those with a small amount of sha should not force the sha; before scraping, the operator should trim the nails to avoid damage to the patient's skin. The strength should be tolerated by the patient, and violence should be avoided; when scraping, you should pay attention to shelter from wind and stay warm. Do not scratch on an empty stomach, excessive fatigue, hypoglycemia, excessive weakness, and nervousness; the scraping board should be used exclusively by special personnel. If conditions do not allow , it needs to be sterilized by high pressure to prevent cross infection; after scraping, the patient should be instructed to drink a cup of warm water, or 200–300 ml of brown sugar water if possible, to promote the discharge of the toxins, and instruct the patient to abstain from cold and greasy food.

### 2.7. Observation Indicators

#### 2.7.1. Comparison of Intervention Effects between the Two Groups

After 2 months of intervention, calculated by nimodipine method; symptom improvement rate = [(total score before treatment—total score after treatment)/total score before treatment] × 100%. Cure, joint pain and swelling disappeared, and there was no significant limitation on motor function or pain or atrophy of small muscles of the hand, or the improvement rate of the main symptoms is 90% or more. Marked improvement, the pain of the joints was relieved, the swelling basically disappeared, the joint movement was slightly restricted, the small muscles of the hands were not obviously atrophied, or the improvement rate of the main symptoms was 70%–89%; Effective, joint pain is slightly improved. There is still swelling. Joint movement is obviously limited. Hand muscle atrophy is not obvious, or the improvement rate of main symptoms is 30%–69%. Ineffective, symptoms did not improve, the range of motion of the shoulder joint was the same as before the treatment, muscle atrophy gradually increased, or the improvement rate of main symptoms was less than 30%. Total effective rate = ((number of cured cases + number of marked improvement cases + number of effective cases)/total number of cases)×100%.

#### 2.7.2. Comparison between the Visual Analogue Scale Score (VAS) and the Degree of Swelling of the Affected Hand before and after the Intervention in the Two Groups

The VAS score was used to evaluate the pain conditions of the two groups of patients before treatment and after 2 courses of treatment. A 10 cm long horizontal line was drawn, with one end being 0 and the other end being 10, indicating different degrees of pain, respectively. Draw a mark on the horizontal line to indicate the level of pain. 0–2 points for comfort, 3-4 points for mild pain, 5-6 points for moderate pain, 7-8 points for severe pain, and 9-10 points for severe pain. Changes in the degree of swelling of the affected hand were graded according to LENT-SOME lymphedema [10]. Grade 1 means that the circumference of the swelling of the upper limb on the affected side is 2–4 cm larger than that of the unaffected limb, and the patient's function is normal; grade II , the swelling circumference of the upper limb on the affected side is 6 cm larger than that of the unaffected limb; grade III is marked thickening of the skin of the entire affected limb and fingers, folds and edema appear, the patient's limb function is severely affected, and the shoulder joint movement is limited. Drainage was recorded by quantifying the difference in drainage volume of the affected hand.

#### 2.7.3. Comparison of Calcitonin Gene-Related Peptide (CGRP) and Substance *p* (SP) Content and Barthel Index before and after Intervention in the Two Groups

Before the intervention and 2 months after the intervention, 3 ml of fasting cubital venous blood was drawn from the patient, centrifuged at 3000 r/min for 10 min, and the serum was separated, placed in an EP tube, and stored in the refrigerator for testing. The serum CGRP and SP contents of patients in each group were detected by enzyme-linked immunosorbent assay. The kits were purchased from Shanghai Zhenke Biotechnology Co., Ltd., and the detection steps were carried out in accordance with the instructions. Barthel index [11]: scores the degree of independence of 10 items of the daily life of patients (eating, bathing, dressing, controlling bowel and bladder, walking on level ground, and going upstairs). Based on a total score of 100 points, it is divided into mild functional impairment, able to complete a part of daily activities independently, and need some help> 60 points. Moderate functional impairment need great help to complete activities of daily living 40–60 points; severe functional impairment, most of the activities of daily living cannot be completed or need help from others 20–39 points; complete disability <20 points.

### 2.8. Statistical Methods

SPSS 22.0 statistical software was used for statistical analysis of the data obtained in this research, and the *χ*^2^ test was used for counting data. The rank-sum test was used for grading data. According to the distribution characteristics of the measurement data, the method is selected, and the measurement data with homogeneity of variance and normal distribution are selected by the *t*-test. Nonparametric tests were used for measurement data that did not conform to the normal distribution. *P* < 0.05 was considered a significant difference, with statistical significance.

## 3. Results

### 3.1. Comparison of Recent Intervention Effects between the Two Groups

After intervention, the total effective rates of the intervention group and the control group were 96.67% and 80.00%, respectively. The total effective rate in the intervention group was significantly higher compared to the control group (*P* < 0.05), as shown in Figure 1.

### 3.2. Comparison of Changes in VAS and the Degree of Swelling of the Affected Hand before and after the Intervention in the Two Groups

After intervention, the VAS score and drainage volume of the two groups of patients were significantly better than those before treatment. The VAS score and drainage volume of the intervention group were lower than those of the control group (*P* < 0.05), as shown in Figure 2.

### 3.3. Comparison of CGRP and SP Contents and Barthel Index before and after Intervention in the Two Groups

After intervention, the CGRP and SP contents and Barthel index of the two groups were better than those before treatment. The CGRP and SP contents of the intervention group were lower than those of the control group, and the Barthel index was higher than that of the control group (*P* < 0.05), as shown in Figure 3.

## 4. Discussion

Stroke is a common neurological disease in my country and even in the world with the rapid onset and severe disease. In recent years, with the development of diagnosis and treatment technology, the mortality rate of this disease has gradually decreased, but the disability rate has shown an upward trend. Among them, shoulder-hand syndrome after stroke, one of the common complications of stroke, is seriously harmful [12]. The onset of shoulder-hand syndrome after stroke varies in priority, which can cause swelling, pain, and severe impairment of motor function in the upper limbs of the patient. If no active treatment is performed, it will cause long-term upper limb dysfunction and even contracture deformities, which will seriously affect the prognosis of patients and quality of life. The effect of scraping mainly depends on the penetration depth of qi and blood, so as to go deep into the viscera and increase the curative effect. The Hufu copper bianstone scraping method is a new technology for poststroke rehabilitation that has been clinically developed and applied in recent years. Hufu copper bianstone is mainly made of copper, and the human body maintains a certain resonance frequency. At the same time, the temperature of the wiping part will also increase to give a warm stimulus. Once the temperature entering the pulse increases, it will be conducive resolving the stasis in the pulse. Besides, the Hufu copper bianstone is rotationally ground on the acupuncture points, so the penetrating power is good, and it is beneficial to transmitting qi and blood to deeper parts [13]. Some studies have confirmed that Hufu copper bianstone scraping can effectively relieve the clinical symptoms of stroke patients [14, 15], but there are relatively few studies on the application of this method to shoulder-hand syndrome after stroke. Therefore, this study will mainly explore the effect of this method on shoulder-hand syndrome after stroke.

Scraping has always been relatively a safe treatment method. During the course of treatment in this study, there were no cases falling off in both groups, and no adverse reactions and complications occurred in the patients, so this point was not highlighted. The results of this study showed that after the intervention, the total effective rates of the intervention group and the control group were 96.67% and 80.00%, respectively. The total effective rate of the intervention group was significantly higher than that of the control group, and the VAS score and drainage volume of the intervention group were lower than those of the control group. This is similar to some research findings [16]. Analysis of the reason is that the Hufu copper scraping bianstone scraping is mainly based on regulating qi, which can mobilize the body's qi and blood activities. The appearance of Sha spots mobilized good recovery ability. Previous studies have shown [17] that the Hufu bianstone is made of copper and can maintain a certain resonance frequency with the human body. At the same time, the temperature of the scraping part will also increase, which has a warming and stimulating effect. The temperature entering the pulse is increased, which is beneficial to resolve the stasis of the pulse. Studies have shown [18] that repeated scraping can promote the production of local stimulants in the skin, accelerate blood circulation, significantly reduce pain, and effectively subside edema. Besides, scraping and grinding can promote vasodilation and rupture, make blood overflow to form ecchymosis, strengthen the body's hemolysis and metabolism, and then resist inflammation. At the same time, it can activate immune cells, strengthen immunity, effectively regulate body functions, and promote the recovery of patients' related symptoms. Above all, it shows that the intervention of Hufu copper bianstone scraping has a significant effect, which can significantly reduce the pain of patients, relieve swelling, and speed up the recovery of patients.

Previous studies have shown [19] that CGRP is a neuropeptide belonging to the calcitonin gene-related peptide family, which is highly expressed in peripheral sensory nerves and the central nervous system, and is involved in the transmission of nociceptive information and the formation of pain sensitization in the periphery and the spinal cord, and interacts with biologically active substances or receptors such as substance P in the process of pain modulation, which has a strong vasodilatory effect. Some studies have shown [20] that the change of CGRP level is related to the severity of nerve damage after hemorrhagic stroke, and it is also an important indicator for evaluating the prognosis of hemorrhagic stroke. The results of this study showed that the content of CGRP in the intervention group was lower than that in the control group after the intervention, indicating that Hufu copper bianstone scraping can effectively promote the recovery of neurological function in patients. SP is a neuropeptide widely distributed in thin nerve fibers. When the nerve is stimulated, SP can be released at the central and peripheral terminals, and can directly or indirectly participate in pain transmission by promoting the release of glutamate, etc., causing nerve neurogenic inflammatory reactions such as vasodilation in the innervation area, increased permeability, and extravasation of plasma proteins, further aggravate the ischemia-hypoxic injury [21]. The decrease of SP level can indicate that the symptoms of county officials in stroke patients can be effectively relieved. The results of this study showed that after the intervention, the SP content of the intervention group was lower than that of the control group, and the Barthel index was higher than that of the control group. Studies have shown that [22], Hufu copper bianstone scraping and grinding the Sanyin and Sanjiao meridians of the hand can stabilize the qi movement and resolve liver qi congestion and blood stasis; Scraping and grinding Dazhui, Dazhu, Gaohuang, Shentang, strengthening the Yang, strengthening the root, strengthening the healthy qi and eliminating the pathogenic factors; Scraping and grinding the acupoints on the head and face, such as Baihui, relax the tendons and activate the collaterals; Scraping the acupoints of the upper limbs can replenish qi so that the qi and blood can reach the end of the body. This method is based on copper for treatment, copper for health, copper for the regulation of liver qi, and copper for the dissipation of wind-phlegm and blood stasis, thereby promoting the recovery of the patient's limb motor function, with few side effects and high safety.

In conclusion, Hufu copper scraping has a significant effect on rehabilitation intervention in patients with poststroke shoulder-hand syndrome, which effectively relieves related symptoms, relieves pain, and promotes the recovery of limb function. It can be used as standardized and effective prevention and treatment method in clinical application.

## Figures and Tables

**Figure 1:** Comparison of recent intervention effects between the two groups. (Note: compared with the control group, ^*∗*^*P* < 0.05).

**Figure 2:** Comparison of the VAS and swelling degree of the affected hands between the two groups before and after intervention (Note: compared with the group before treatment, ^*a*^*P* < 0.05; compared with the control group, ^*b*^*P* < 0.05).

**Figure 3:** Comparison of CGRP, SP content, and Barthel index between the two groups before and after the intervention (Note: compared with the group before treatment, ^*a*^*P* < 0.05; compared with the control group, ^*b*^*P* < 0.05).

## Data Availability

The data to support this study are available from the corresponding author upon request.
